# Galectin-1, -4, and -7 Were Associated with High Activity of Disease in Patients with Rheumatoid Arthritis

This article has been retracted.

**DOI:** 10.1155/2019/3081621

**Published:** 2019-07-22

**Authors:** Kamila de Melo Vilar, Michelly Cristiny Pereira, Andrea Tavares Dantas, Moacyr Jesus Barreto de Melo Rêgo, Ivan da Rocha Pitta, Claudia Diniz Lopes Marques, Rafaela Silva Guimarães Gonçalves, Laurindo Ferreira da Rocha Júnior, Ângela Luzia Branco Pinto Duarte, Maira Galdino da Rocha Pitta

**Affiliations:** ^1^Laboratory of Immunomodulation and New Therapeutic Approaches (LINAT), Suely-Galdino Therapeutic Innovation Research Center (NUPIT-SG), Federal University of Pernambuco (UFPE), Recife, PE, Brazil; ^2^Rheumatology Service, Clinical Hospital, UFPE, Recife, PE, Brazil; ^3^Laboratory for Planning and Synthesis of Drugs (LPSF) of the Federal University of Pernambuco (UFPE), Recife, PE, Brazil

## Abstract

**Background:**

Due to the variety of functions that galectins (Gal) possess, it is clear that they participate in the pathogenesis of rheumatoid arthritis (RA). Although some studies demonstrate their functions, there is still no correlation with the clinical data of the disease, having the physiological meaning still unknown.

**Objectives:**

To compare serum levels of Gal-1, -4, and -7 in patients with RA and healthy controls and to correlate them with clinical parameters.

**Methods:**

Serum samples were collected from patients with RA and healthy donors to determine the serum levels of Gal-1, -4, and -7.

**Results:**

Serum levels of Gal-1, -4, and -7 were significantly higher in RA patients compared to controls. We evaluated disease activity (CDAI) with serum levels of galectins and found that patients who were high in disease activity had high levels of galectin compared to the moderate activity group. Galectin-4 had higher levels in patients who were in high activity when compared to the group in remission or low activity. Evaluating the activity of the individual disease (DAS28), patients in high individual activity had high levels of Gal-4 when compared to the group in remission or low activity. We also found an association between positive rheumatoid factor and Gal-1 and Gal-4 levels.

**Conclusion:**

Our results show for the first time the relationship between serum levels of galectin and the clinical parameters of patients with RA. Demonstrating their role in pathogenesis, new studies with galectins are needed to assess how they function as a biomarker in RA.

## 1. Introduction

Rheumatoid arthritis (RA) systemic autoimmune disease, characterized persistent synovial inflammation, and associated damage to articular cartilage and underlying bone are present [1]. According to the World Health Organization (WHO), RA affects adults, reaching one in every 100 people, with a higher prevalence in women. In Brazil, it is estimated that the prevalence of RA ranges from 0.2 to 1% and presents worldwide distribution [2, 3]. Genetic and environmental factors contribute to the development. Environmental risk factors such as bacterial and viral infections, smoking, and alcohol consumption are also related to the pathogenesis of the disease [4, 5].

The autoimmune response in RA is the presence of autoantibodies, especially those directed to immunoglobulin G, rheumatoid factor (RF), and citrullinated peptides (ACPA), causing infiltration of multiple leukocytes in the joints, including B cells, T cells, macrophages, dendritic cells, and neutrophils [6]. The presence of autoreactive T and B cells leads to synovitis and cell infiltration, causing a process of bone destruction and remodeling. CD4^+^ T cells are the dominant T-cell types in the synovium, Th17, being a subset of helper T cells secreting interleukin-17 (IL-17) with overproduction and overexpression of tumor necrosis factor alpha (TNF-*α*) causing the destruction of regulatory T cells (Treg). This process leads to overproduction of many cytokines, such as IL-6, IL-1, which also drives persistent inflammation and destruction of the joints, playing a critical role in pathogenesis [7, 8]. In addition, the recognition of immune complexes by phagocytes promotes the release of several proinflammatory cytokines, especially TNF-*α*, which further increases the inflammatory process [8].

The family of galectins is involved in a wide range of biological processes and has been detected in numerous tissues and organs, having an important role in the pathophysiology of diverse diseases, including RA [9]. Galectins are lectins that specifically bind to *β*-galactoside carbohydrates at the cell surface or in the extracellular space and share significant sequence similarity in their carbohydrate-recognition domains (CRDs) [9, 10]. To date, at least 15 galectins have been identified, all of which contain one or two CRDs of about 130 amino acids each. Based on the CRD organization, galectins are divided into three subfamilies: the “prototype” subfamily that contains only one CRD (galectin‐1, ‐2, ‐5, ‐7, ‐10, ‐11, ‐13, and ‐14); the “tandem‐repeat type” subfamily that has two separate CRDs connected by nonconserved amino acid sequences (galectin-4,-6, -8, -9, and -12); and the “chimeric-type” subfamily contains one CRD and a nonlectin region of about 120 residues at the N-terminal of CRD (galectin-3) [11, 12]. These lectins have been detected in numerous tissues and organs. Due to the absence of the classical signal sequence for incorporation into the endoplasmic reticulum (ER), they primarily localize intracellularly; some types of galectins can be found on the cell surface with galectin-9 or secreted through a nonclassical ER/Golgi-independent pathway to the extracellular compartment with galectin-1 and -3 [13].

Galectin-1 is a member of “prototype” that has a special affinity for* N*-acetyllactosamine residues on extracellular glycoproteins. This galectin has a key role in the regulation of the immune system and oncogenesis [14]. There is a potent apoptotic effect of galectin-1 on activated T cells, where surface molecules CD7, CD43, and CD45 exist. Regarding its effect on the immune response, galectin-1 seems to have a strong effect modulating the inflammatory response, suggesting a potential therapeutic use [15, 16]. In RA, Gal-1 levels were significantly reduced in synovial fluid in patients, possibly due to the increase of anti-Gal-1 autoantibodies limiting the amount Gal-1 and potentially blocking its biological effect in patients with RA [17].

Galectin-4 is a member of “tandem-repeat type” having the characteristic of specifically binding to *β*-galactosides through the two structurally conserved CRDs. Due to its bivalent or multivalent structure, galectin-4 plays an important role in biochemical regulation and tumor development and progression [18]. Due to the lack of signal sequence for the transport of ER, the presence of galectin-4 on the cell surface is a consequence of secretion via the nonclassical pathway; thus, intracellular galectin-4 regulates cell proliferation, apoptosis, and differentiation, while extracellular galectin-4 mediates intercellular adhesion [19, 20]. Its role is well studied in cancer and inflammatory bowel diseases, such as Crohn's disease (CD) and ulcerative colitis (UC), where there is an activation of inflammatory memory CD4^+^ T cells in the inflamed gastrointestinal tract [20]. However, to date, there are no studies demonstrating the role of this galectin in autoimmune diseases, especially in rheumatoid arthritis.

Galectin-7 appears to preferentially bind to the internal or terminal LacNAc repeat carried out by the N-glycan and as additional prototypic component is capable of forming homodimers through a back-to-back arrangement, resulting in an interface of greater magnitude compared with other prototypic galectins [21]. This difference in structural arrangement suggests that galactin-7 glycoconjugate binding activity may differ from other prototypical ones. So galectin-7 participates in diverse processes such as the susceptibility to apoptosis, cell migration, and cell adhesion and has been in stratified epithelia where it favors epithelial homeostasis [22, 23]. To date, there are no studies demonstrating galectin-7 function in RA.

Because of the diversity of functions of galectins, the objective of this study was to evaluate the serum levels of Gal-1, Gal-4, and Gal-7 in patients with rheumatoid arthritis correlating with clinical data in order to find a possible biomarker of the disease.

## 2. Materials and Methods

### 2.1. Study Population

A total of 229 patients with RA (220 women, 9 men; mean age 52.66 yrs) were recruited from the Department of Rheumatology at Hospital das Clínicas da Universidade Federal de Pernambuco (UFPE). The diagnosis of RA was established by the American College of Rheumatology 1987 diagnostic criteria [24]. About 170 healthy volunteers (137 women, 33 men; mean age 49.57 yrs) were included as controls, and all were free of any rheumatologic conditions. Peripheral blood samples were obtained from patients and controls. Demographic, clinical, and laboratory data were collected from hospital records or by questionnaire and reviewed by experienced physicians.  Table 1 presents demographic and clinical findings in patients with RA and laboratory features of patients with RA erythrocyte sedimentation rate (ESR), rheumatoid factor (RF). Individual disease activity was quantified using the Disease Activity Score for 28 joints (DAS28) [25] and the Clinical Disease Activity Index (CDAI) [26]. Radiographs of hands were obtained from patients with RA and evaluated for the presence of erosions by an experienced rheumatologist blinded to the clinical data. The study was approved by the ethics committee of the UFPE (CAAE: 63648616.0.0000.5208).

### 2.2. Measurement of Serum Galectins Levels

Galectins in serum were assayed with an ELISA kit according to the manufacturer's recommendation (R&D Systems). The lower limit of detection for the ELISA galectin-1 kit was 156.25 pg/ml, galectin-4 was 15.625 pg/ml, and galectin-7 was 78.125 pg/ml.

### 2.3. Statistical Analysis

Associations of serum of galectins levels with clinical and laboratory measures of patients with RA were analyzed by univariate comparisons using nonparametric tests (Mann-Whitney tests). p < 0.01 was considered a significant association and p < 0.05 a suggestive association. Results are shown considering the mean value. All quantitative data were plotted with GraphPad Prism 6.0 software.

## 3. Results

The basic characteristics of the study subjects are shown in Table 1. Galectin levels were detected in patients when compared to the control group (Gal-1: p <0.0001, median= 5435 pg/ml; Gal-4: p <0.0001, median=702.30 pg/ml; and Gal- 7: p <0.0001, median=2134 pg/ml) (Figure 1). We evaluated the levels of galectins in relation to the clinical activity of the patients. Patients who presented moderate disease activity (CDAI: 10>,  <22) were associated with higher levels of Gal-1 when compared to patients in remission or low moderate activity (CDAI: <10) (p = 0.0263, median= 3673 pg/ml). Patients who had high activity (CDAI: >22) also had high levels of Gal-1 when compared to the group in remission or low disease activity (CDAI: <10) (p = 0.0476, median= 3210 pg/ml) (Figure 2(a)). We did not find any correlation between the levels of Gal-7 and the parameters of disease activity.

We also observe that patients who were in moderate activity (CDAI: 10>,  <22) had high levels of galectin-4 when compared to those in remission or low activity (CDAI: <10) (p = 0, 0117, median = 518.9 pg/ml) (Figure 2(b)). High levels of Gal-4 were also found in patients with high activity (CDAI: > 22) when compared to the group in remission or low activity (CDAI: <10) and high activity (p <0.0001, median= 346,0 pg/ml) (Figure 2(b)). Patients with moderate individual activity (DAS28: 3.2>,  <5.1) presented high levels when compared with patients in remission (DAS28: <3.2) (p = 0.0280, median= 587.3 pg/ml) (Figure 3). Patients in high individual activity (DAS28: > 5.1) had high levels of Gal-4 when compared to the group in remission or low activity (DAS28: <3.2) and moderate individual activity (DAS28: 3.2<5.1) (p <0.0001, median= 391.0 pg/ml; p = 0.0012, median= 391.0 pg/ml, respectively) (Figure 3). Evaluating rheumatoid factor (RF), patients with positive RF had higher levels of Gal-1 and Gal-4 compared to negative patients, respectively, p = 0.0358, median= 7057 pg/ml; p = 0.0099, median= 864.1 pg/ml (Figures 4(a) and 4(b)).

## 4. Discussion

Galectin-1 has been shown to be an important modulator of cell homeostasis by inducing apoptosis in different cell types, such as monocytes and cells, in addition to cell survival and proliferation [27, 28]. Previous studies have suggested a possible therapeutic effect after the application of Gal-1 in rat with RA models [17, 29], while another study has shown that galectin-1 expression has been downregulated in juvenile idiopathic arthritis characterized by synovial cell hyperplasia; however, its implication in the physiology of human disease remains unknown [30, 31]. Our current results show a significant increase in patients with RA compared to control (p<0.0001) (Figure 1). It is well known Gal-1 levels markedly increase in sera from RA patients and positively correlate with an erythrocyte sedimentation rate (ERS) and disease activity score 28 (DAS-28) parameters [17]. The activity indexes that are available and recommended for use in clinical trials comprise the DAS28, the simplified disease activity index (SDAI), and CDAI [32]. Synovial proteome studies have confirmed the presence of Gal-1 in patients with RA, suggesting increased inflammatory role compared to osteoarthritis patients [30, 33]. Our findings corroborate previous studies since serum levels of this galectin are present in greater numbers in our group of patients with remission of disease (p = 0.0476) (Figure 2(a)). Laboratory tests were also related to serum levels of Gal-1 in patients. Patients who presented with positive rheumatoid factor, whose presence suggests a worse prognosis of the disease, had high levels of galectin (p = 0.0232) (Figure 4(a)). A recent study demonstrated the role of gal-1 in RA, where high levels of this galectin were found in patients, in addition to the association of gal-1 with disease activity indicating that galectin may contribute to the anti-inflammatory effects caused by DMARDs and corticosteroid therapy in patients with RA [17]. Thus, although its function is not completely understood, our results corroborate with the findings of the literature suggesting that the presence of this galectin is related to the worse prognosis of the disease.

Galectin-4 is an important lectin-related to mucosal immunity and is strongly associated with increased intestinal inflammation by directly stimulating CD4^+^ T cells to produce IL-6 in the TCR mutational colitis model [34]. IL-6 is a cytokine with a proinflammatory activity that affects both the innate and adaptive immune system, which is present in the pathogenesis of rheumatoid arthritis [35]. Through an immunological synapse linkage, which occurs through a specific activator of the signaling cascade associated with protein kinase C (PKC), Gal-4 can interact with CD4^+^ T cells stimulating IL-6 production causing an increase in inflammation intestinal. However, studies have shown that galectin-4 can induce T-cell apoptosis through its binding to the CD3 epitope, which is present on the T-cell surface in the wild-type colitis model. Once such binding occurs, the complex formed promotes apoptosis of T cells in a calpain-dependent manner and a reduction of cytokine secretion, including IL-6, leading to an improvement in inflammation [19, 36]. To date, the implication in the physiology of autoimmune disease remains unknown. Thus, our result presents unprecedented evidence that Gal-4 is present at high levels compared to controls (p <0.0001) (Figure 1). Regarding the clinical parameters, high levels of Gal-4 were found in patients with high activity (CDAI: >22) when compared to the group in remission or low activity (CDAI: <10) (p <0.0001) (Figure 2(b)). The individual activity of the disease (DAS28) evaluated in patients with high individual activity (DAS28:> 5.2) had high levels of Gal-4 when compared to the group in remission or low activity (DAS28: <3.2) and moderate individual activity (DAS28: 3.2 < 5.1) (p <0.0001, p = 0.0012, respectively) (Figure 3). Positive rheumatoid factor was also associated with high levels of Gal-4, which corroborates the above results (p=0.0013) (Figure 4(b)). Since several mechanisms may be related to the development and worse prognosis of the disease, the presence of galectin-4 may clarify the mechanism of RA somewhat, since patients with high disease activity are related to Gal-4 levels suggesting that their presence may be related to the worst prognosis of the disease. New studies must be carried out to define the role of this Gal-4 in RA pathogenesis.

Galectin-7 has several cellular functions, most of them related to the maintenance of epithelial integrity, induction of apoptosis of activated T cells with an of caspase activation, and also acts as antifibrotic factors liver fibrosis [37, 38]. A previous study evaluated the serum of patients with various autoimmune diseases for autoantibodies, where the response profile characterizes the type of disease. The findings suggest that autoantibodies present in serum may contribute to dysregulation of the immune system, where the immunological response to age and sex in the controls was found against the Gal-7 prototype, with indications for Gal-7 positivity in patients with systemic lupus erythematosus. In addition to the presence of autoantibodies, galectin-2, -3, -4 and -7 were highly significant in arterial and venous thrombosis, recurrent miscarriages, and thrombocytopenia [39]. To date, there is no data demonstrating a relation between Gal-7 and RA. Our results are unprecedented in demonstrating for the first time that RA patients have high levels of Gal-7 compared to controls (p <0.0001) (Figure 1). However, we did not find positive associations regarding the parameters of disease activity. More studies are needed to demonstrate its true role in this disease.

## 5. Conclusion

Our results show for the first time the relationship between serum levels of galectin and the clinical parameters of patients with RA, demonstrating for the first time in the literature the role of galectin-4 and galectin-7 in rheumatoid arthritis, in addition to the correlations of galectin-1 and -4 with clinical data of the patients. High levels of these galectins are related to patients in high activity and the presence of rheumatoid factor. In this way, galectin can act as the biomarker of the disease. Further studies must be performed to confirm the results.

## Figures and Tables

**Figure 1:** Comparison of the serum levels of galectin-1, -4, and -7 in the patients and controls (p<0.0001).

**Figure 2:** (a) Evaluation of Clinical Disease Activity Index with serum levels of Galectin-1. (b) Evaluation of Clinical Disease Activity Index with serum levels of galectin-4.

**Figure 3:** Evaluation of the Disease Activity Score for 28 joints (DAS28) with serum levels of galectin-4.

**Figure 4:** (a) Evaluation of rheumatoid factor and levels of Galectin-1. (b) Evaluation of rheumatoid factor and levels of galectin-4.

**Table 1:** Demographic and clinical parameters of RA patients and control population.

*N*umber of *Controls*	170
Female/male	137/33
Mean age (min-max)	49.44 (19-82)

*N*umber *of patients*	229
Female/male	220/9
Mean age	52.66 (18-78)

*Disease Activity Score 28 joints (%)*	
Clinical remission	114 (49.78)
Moderate disease	70 (30.56)
Severe disease	45 (19.65)

*CDAI (*%)	
Clinical remission	158 (68.99)
Moderate disease	40 (17.46)
Severe disease	31 (13.53)

*HAQ*	
<1	64 (27.94)
>1	121 (52.83)

*Rheumatoid factor (*%)	
Positive	130 (56.76)
Negative	76 (33.18)

*Radiological erosions (*%)	
Present	101 (44.10)
Absent	74 (32.31)

*Erythrocyte sedimentation rate (ESR – mm/h)*	33.01 (0-125)

## Data Availability

The patient's data used to support the findings of this study are restricted by the research ethics committee in order to protect patient privacy. Data are available from Maira Pitta (mgrpitta@gmail.com) for researchers who meet the criteria for access to confidential data.
